# Polymorphism of C3 complement in association with myocardial infarction in a sample of central Tunisia

**DOI:** 10.1186/1746-1596-8-93

**Published:** 2013-06-13

**Authors:** Nadia Leban, Karim Jraba, Abdelkader Chalghoum, Selma Hassine, Donia Elhayek, Sabri Denden, Ramzi Lakhdhar, Faouzi Maatoug, Habib Gamra, Hammadi Braham, Jemni Ben Chibani, Amel Haj Khelil

**Affiliations:** 1 Biochemistry and Molecular Biology Laboratory, Faculty of Pharmacy, Street Avicenne, 5019 Monastir, Tunisia; 2 Cardiology Department, Fattouma Bourguiba Universitary Hospital, Monastir, Tunisia; 3 Biochemistry and Blood Bank Department, Universitary Hospital Taher Sfar, Mahdia, Tunisia

**Keywords:** Myocardial infarction, C3 complement, Polymorphism, Allele frequency, Association

## Abstract

**Background:**

Myocardial infarction (MI) is a major clinical problem because of its large contribution to mortality. The genetic bases of this disease have been widely studied in recent years to find a clear association with some genetic markers that increase the risk of its occurrence. In the present investigation, the correlation between MI and the C3 complement polymorphism was analyzed using a case–control study.

**Methods:**

Our study ported on one hundred seventy survived myocardial infarction patients and ninety five healthy controls. The C3 allele identification was investigated using the amplification refractory mutation system PCR to determine the C3*S and the C3*F alleles of the C3 polymorphism.

**Results:**

Frequencies of C3*S and C3*F in patients are 0.59 and 0.41 respectively. Fisher test results showed a significant increase of C3*F allele in the sample of patients (0.41; odds ratio: 2.616; C.I [1.738-3.938]) compared to controls (0.21; odds ratio: 0.382; 95% CI [0.254-0.575]), p = 2.742 × 10^-6^.

**Conclusion:**

A strong positive correlation was found between C3 polymorphism and MI estimating that the risk of myocardial infarction is significantly increased among patients with C3*F allele of this polymorphism.

**Virtual Slides:**

The virtual slide(s) for this article can be found here: http://www.diagnosticpathology.diagnomx.eu/vs/1190484203893646

## Introduction

Myocardial infarction (MI) is the rapid development of myocardial necrosis caused by a critical imbalance between oxygen supply and demand of the myocardium. This usually results from plaque rupture with thrombus formation in a coronary vessel, resulting in an acute reduction of blood supply to a portion of the myocardium. Important risk factors are: previous cardiovascular disease, older age, tobacco smoking, high blood levels of certain lipids (triglycerides, low-density lipoprotein) and low levels of high density lipoprotein (HDL), diabetes, high blood pressure, obesity, chronic kidney disease, heart failure, excessive alcohol consumption, abuse of certain drugs, Thiamine deficiency (beriberi), and chronic high stress levels [1-3]. MI is a major clinical problem because of its large contribution to mortality. According to the World Health Organization, heart attacks are among the most important cause of death for both men and women all over the world.

In addition to these common risk factors, studies have shown the importance of genetic factors. The genetic bases of this disease have been widely studied to find a clear association between the MI and some genetic markers that increase the risk of its occurrence (Table 1). Among the studied genetic markers we find the C3 component of the complement. The C3 protein is composed of 1663 amino acids. The C3 gene is localized in 19 p13.3-2 and contains 41 exons spread over 41 Kb. The polymorphism of the C3 gene is under the control of codominant autosomal alleles. The two most common allotypes are C3*S (S for slow) and C3*F (F for fast). The C3 polymorphism (R102G) consists on G to C substitution at position 364 in exon 3 leading to a change of Arginine in C3*S to Glycine in C3*F [4].

**Table 1:** List of genetic markers analyzed for the association with myocardial infarction

**Gene**	**Polymorphism**	**Association**	**References**
C3 complement	C3*S	-	[5,6]
	C3*F	+	[7]
CYP2J2	G50T	-	[8]
VEGF	−634	+	[9]
COX-2	PTGS2	+	[10]
PGIS	CYP8A1	+	
IL-18 promoter	−607C/A	+	[11]
	−137 G/C	-	
PSMA6	−8C > G	+	[12]
MTAP	21807754 G/A	+	[13]
CDKN2B	21993223 G > A	+	
	21993367 A/G	+	
Fas promoter	−670 G/A	+	[14]
Serotonin transporter	5-HTTLPR (L/S)	+	[15]
ACE	Insertion/Deletion	+	[16]
Near INSIG2	7543947C > G	-	[17]
MCP-1	−2518A > G	-	[18]

(+): positive; (−): negative.

The C3 complement component polymorphism was often used as a powerful marker for genetic studies of populations [19], since it is biallelic and codominant single nucleotide polymorphism, the complement system has a critical role in both the innate and the adaptive immune responses [20]. In humans, C3*F (C3102G) has been associated with autoimmune diseases [21,22]. Few researches are carried out in the literature on the correlation between C3 polymorphism and MI. This relationship has been studied most often on the serum level. Previous studies showed that the C3 serum protein is correlated with a set of risk factors for MI [23]. Considering the pathophysiological data, it seems that the carriers of the C3*F allele are able to control inflammatory diseases to a lesser extent than non-carriers may do. Therefore, in the case of C3*F carriers, there may be a higher likelihood of inflammation within the vulnerable plaques that may facilitate their rupture [24] and the consequential development of myocardial infarction. The more common C3*S allele may have an effect of opposite direction that protects against the development of MI [7]. C3 could be considered as a factor screening primary prevention of myocardial infarction [25]. In this context, we are interested to analyze the association between the single-nucleotide polymorphism in the C3 complement component gene and the risk of developing MI in the Tunisian population. To achieve this purpose, we carried out a case control study. This research falls within the framework of improving the strategy for prevention of this disease. By identifying the genetic markers that may increase the risk of its occurrence, it would be possible to carry out the interventions needed to reduce the possibility of future events.

## Methods

### Study populations

This work was performed on 170 blood samples of patients aged between 44 and 83 years (mean age: 65,48 ±10,91 years) who have survived to myocardial infarction followed in the cardiology departments at the University Hospitals of Sousse, Monastir and Mahdia. For blood collect, we have obtained approval from the Hospital authority and the ethics committee after consent of patients. For each patients, we reported the body mass index, the triglycerides, HDL-c, LDL-c and cholesterol concentrations, the risk factors (mainly smoking), and the history of the disease (such as diabetes, arterial hypertension, dyslipidemia,…). Ninety-five healthy Tunisian adult blood donors were included in the study as control sample.

### Genetic analysis

DNA extraction was performed on 5 ml of peripheral-blood samples collected on EDTA from patients and controls using the standard phenol/chloroform method. Amplification Refractory mutation System (ARMS) PCR [26] was used for the two groups to determine the C3*S and C3*F alleles. The technique requires that the terminal 3'-nucleotide only of a PCR primer be allele specific. Thus the primer is synthesized in two forms. The normal form (C3*S primer) is refractory to PCR on mutant template DNA (C3*F) and *vice versa*. Introducing additional deliberate mismatches near the 3' end of appropriate primers does not allow non specific amplification to proceed, that’s why we preferred this method which seems more convenient for genotyping than enzymatic digestion which requires two reactions to be performed.

In the ARMS reaction, three primes were used: one common reverse primer (5′-TGTTGACCATGACCGTCCGGCCCACGGTA-3′) and two forward specific primers (5′-CCAACAGGGAGTTCAAGTCAAAAGGTGG-3′ for C3*S and 5′-CCAACAGGGAGTTCAAGTCAGAAAAGGTGC-3′ for C3*F). For each DNA, the amplification is performed twice on a final volume of 25 μl containing 100 ng of DNA, 0.6 μM of each primer, 3 mM of MgCl_2_, 0.32 mM of each dNTP and 1.5 U of Taq polymerase (Promega). The reaction is performed on an Appligene Oncor thermocycler under the following conditions: 2 min at 94°C, 33 cycles of 30 s at 94°C, 1 min at 50°C, 1 min at 72°C and finally, one cycle of 10 min at 72°C. PCR products were revealed on 2% agarose gel electrophoresis and visualized under UV light after ethidium bromide staining. Genotypes are determined for all individuals and frequencies are calculated for the two alleles.

### Statistical analysis

Allele frequencies are compared in the samples of MI patients and controls using Epi info 6 software (Fisher test).

## Results

The ARMS PCR allowed to determine the different genotypes since homozygous DNA for C3*F and C3*S alleles are amplified only in presence of F or S specific primers respectively whereas heterozygous DNA are amplified in presence of both primers (Figure 1). The genotyping of MI samples allowed calculating the allelic frequencies of C3 under the hypothesis of Hardy-Weinberg equilibrium. Results for the equilibrium test showed that the difference between observed and expected frequencies is not significant (χ^2^ = 1.286 < 3.84).

**Figure 1:** Molecular identification of C3*S and C3*F alleles by agarose gel electrophoresis of ARMS-PCR products (318 bp fragment). M: molecular weight ladder (100 bp); 1: negative controls; 2: positive controls; 3;…,8: analyzed DNA; S: C3*S specific PCR product; F: C3*F specific PCR product. Genotypes: 3: SS; 4: SF; 5: SS; 6: FF; 7: SS.

The genotype and alleles frequencies of C3*S and C3*F found in this study are summarized in Table 2. These values are compared with those of controls.

**Table 2:** Association test between C3 polymorphism and myocardial infarction by comparing genotype and allele frequencies of C3*S and C3*F in patients and controls

		**Controls**	**MI patients**	**Fisher test**	
**Number**		**95**	**170**		
**Allelic Frequencies**	C3*S	0.79	0.59	Odds ratio = 0.382	p = 2.742 × 10^-6^
				C.I. = [0.254-0.575]	
	C3*F	0.21	0.41	Odds ratio = 2.616	
				C.I. = [1.738-3.938]	

CI: confidence interval, MI: myocardial infarction.

C3*S allele frequency is higher than C3*F in the two populations (controls and patients). For the C3*F allele, the frequency found in patients (0.41) is 2 times higher than that found in controls (0.21). Thus, the C3*S allele frequency is reduced (0.59) in the sample of patients compared to that of controls (0.79).

Fisher test results showed a significant increase of C3*F allele in the sample of patients (p = 2.742 × 10^-6^). Therefore, it is estimated that the risk of myocardial infarction is significantly increased among patients with the C3*F polymorphism (Table 2).

## Discussion

Our results about the allelic frequencies of the donors sample are compared to those of previous study in which sera from 95 healthy donors (representative of the Tunisian general population) are phenotyped using agarose gel electrophoresis [27]. The similarity observed between C3*S and C3*F frequencies in the two studies strengthens our findings.

Our results showed a strong association between C3*F polymorphism and the risk of the MI since the probability P is 2.742 × 10^-6^ (<0.05). Based on these results, homozygous for the C3*S allele are more protected against the occurrence of myocardial infarction. In the contrary, this risk is highly increased for homozygous C3*F individuals.

In the literature, only few associations between the C3 component polymorphism and myocardial infarction have been analyzed. In one of them, carried out on the territory of Delhi (India), the difference between MI cases and controls was found to be statistically non-significant indicating that, in this Indian population, the C3 marker is not associated with the risk of myocardial infarction [6]. Another study was a C3 phenotype serum investigation in patients with heart infarct. Despite differences in the percentage distribution of various phenotypes between the patients’ sera and those of controls, no significant association could be established [5]. However, a positive correlation was found in the Hungarian population in which the C3*F allele may be associated with an increased risk of developing myocardial infarction in coronary heart disease patients [7].

Several associations of the C3 polymorphism with other diseases have been reported (Table 3). Atherosclerosis is an inflammatory disease and the complement system plays an important role in its process. Previous study provides further evidence of a positive association of the C3*F allele with atherosclerosis, and it is concluded that this allele in a hypertensive patient might accelerate the atherosclerotic process, with subsequent premature development of vascular complications [28]. Significantly increased frequency of C3*F was observed in patients with the cardiomyopatic form of Chagas disease compared to those presenting the asymptomatic indetermined form and with the healthy controls. These results present the C3*F allele as a susceptible marker for the progression of the cardiomyopatic form of Chagas disease [29]. Further investigations showed a significant risk of lung cancer among men of the C3 SF/FF genotypes compared to the SS genotype [30]. Finally, many studies have demonstrated an association between the C3*F allele and the presence of age-related macular degeneration (AMD) [31-33].

**Table 3:** Association of C3 polymorphism with various cardiopathies

**Disease**	**Allele frequencies**						**References**
	**Controls**			**Patients**			
	**N**	C3*S	C3*F	**N’**	C3*S	C3*F	
**Cardiomyopathy**	100	0.840	0.160	57	0.771	0.228*	[33]
**Coronary heart disease (CHD)**	523	0.832	0.168	171	0.827	0.213*	[7]
**Atherosclerosis**	62	0.882	0.118	139	0.532	0.468*	[32]

N and N’: number of individuals, *: significant difference (P < 0.05).

### How explain the implication of the variant C3F in the diseases development?

Number of studies suggests that functional differences exist between C3 complement allotypes F and S in the pathogenesis of MI and other diseases with a higher risk found in individuals with allotype F. Hemolytic activity is slower for C3*F than for C3*S products [34]. It has been shown that erythrocytes encoded with C3*F are surrounded by much more bearing monocytes than C3*S [35].

The C3F variant bound Factor H Complement (CFH) less than C3S, causing decreased Factor I Complement cofactor activity, and enhanced C3 alternative pathway amplification. By combining risk and protective alternative pathway variants (activators and regulators), it has been shown that C3, CFH, and Factor B variants collaborate to set levels of alternative pathway of systemic complement activity in plasma, thereby influencing risk in complement-dependent diseases [36]. However, no difference between C3*F and C3*S forms in their binding to complement receptors types 1, 2 and 3 was shown [37]. In addition, in vitro experimental evidence showing functional differences between the two forms of C3 is not conclusive [31].

## Conclusion

In conclusion, our study showed a strong association between the C3*F variant and MI, (0.41 versus 0.21 with p = 2.742 × 10^-6^). C3*F appears to have a causal role in increasing the risk of occurrence of this disease. These results add to our understanding of the genetic factors of myocardial infarction and provide evidence that the C3 complement component may be a predisposing factor for this common disease. The determination of C3 polymorphism may help in the identification of patients at risk for developing MI.

## Competing interests

The authors declare that they have no competing interests.

## Authors’ contributions

All authors read and approved the final manuscript.
